The article "Spoken Language Identification Using Deep Learning" was published in 2021. Journal: Comput Intell Neurosci.

# Spoken Language Identification Using Deep Learning

**DOI:** 10.1155/2021/5123671

**Published:** 2021-09-20

**Authors:** Gundeep Singh, Sahil Sharma, Vijay Kumar, Manjit Kaur, Mohammed Baz, Mehedi Masud

**Affiliations:** ^1^Computer Science and Engineering Department, Thapar Institute of Engineering and Technology, Patiala, India; ^2^Computer Science and Engineering Department, National Institute of Technology, Hamirpur, India; ^3^School of Engineering and Applied Sciences, Bennett University, Greater Noida, India; ^4^Department of Computer Engineering, College of Computer and Information Technology, Taif University, P.O. Box. 11099, Taif 21994, Saudi Arabia; ^5^Department of Computer Science, College of Computer and Information Technology, Taif University, P.O. Box. 11099, Taif 21994, Saudi Arabia

## Abstract

The process of detecting language from an audio clip by an unknown speaker, regardless of gender, manner of speaking, and distinct age speaker, is defined as spoken language identification (SLID). The considerable task is to recognize the features that can distinguish between languages clearly and efficiently. The model uses audio files and converts those files into spectrogram images. It applies the convolutional neural network (CNN) to bring out main attributes or features to detect output easily. The main objective is to detect languages out of English, French, Spanish, and German, Estonian, Tamil, Mandarin, Turkish, Chinese, Arabic, Hindi, Indonesian, Portuguese, Japanese, Latin, Dutch, Portuguese, Pushto, Romanian, Korean, Russian, Swedish, Tamil, Thai, and Urdu. An experiment was conducted on different audio files using the Kaggle dataset named spoken language identification. These audio files are comprised of utterances, each of them spanning over a fixed duration of 10 seconds. The whole dataset is split into training and test sets. Preparatory results give an overall accuracy of 98%. Extensive and accurate testing show an overall accuracy of 88%.

## 1. Introduction

Spoken language identification (SLID) is recognizing the language being a talk by an anonymous speaker from an audio clip. Humans are the most error-free language identification system [1]. There are various implementations of spoken language identification like creating front ends for multilanguage speech identification systems, automatic customer routing in call centers, monitoring, and web information retrieval [2]. The SLID system has three main parts, data collection, feature removal, and language classification, as shown in Figure 1. An essential for developing and evaluating a speech recognition system is the accessibility of a suitable database [3].

Different methods have been proposed to figure out the problems of automatic language identification with the acoustic phonetics approach [1, 4]. Encouragement in the deep learning field has empowered researchers to use GANs for language identification for robustness on unsupervised and semisupervised tasks [5]. Support vector machines (SVM) classifiers do not work well on short utterances, giving less accuracy [6]. Conventional identification systems are supported on i-vector systems for spoken language processing tasks, which are inefficient [7].

To resolve the problems which are mentioned above, a log-Mel spectrum is used to generate the spectrograms of audio snippets, which can record or store the frequency of particular audio utterances. It is efficient and fast, and further, we can apply the convolutional neural network (CNN) technique to classify different languages. This work has been done using the spectrum technique using deep learning by the authors [8]. Many researchers are working on image creations and image identification using a deep learning technique that gives good results and better accuracy in 2D [9, 10], 2.5D [11], and 3D [12, 13] domain. There is a challenge to identify spoken language with different genders, other age groups, and various accents. There is noise in the background in some of the audio clips, so it is very hard to identify the language. A deep learning CNN technique is proposed to draw out the attributes.  Figure 2 shows the phases of the proposed spoken language identification framework. A prediction is made by a model, which can easily identify classification in the proposed framework.

1. A novel deep learning-based model is proposed to apply the convolutional neural network (CNN) to draw out attributes from images.
2. The proposed model is analyzed with different deep learning and machine learning techniques over four datasets.
3. The proposed approach differs from other state-of-the-art methods on various evaluation metrics and shows the comparison with different techniques.

The formation of work is as follows: Section 2 represents an explorative concept of spoken language identification using CNN.  Section 3 discusses past studies in the language identification field.  Section 4 discusses the model architecture of raw waveforms and log-Mel spectrogram images.  Section 5 represents an experimental result. In Section 6, consequences and results are discussed. Finally, Section 7 concludes the paper.

## 2. Background

This section discusses the preliminary concepts of spoken language identification using CNN, spectrograms, and Multinomial Naïve Bayes.

### 2.1. Spoken Language Identification Using CNN

The process of spoken language identification using the CNN technique uses spectrograms of raw audio signals as input to a convolutional neural network (CNN) [8, 14]. A spoken language identification dataset is collected and preprocessed for the training phase. The main focus is on preprocessing, in which we convert audio utterances in spectrogram images. After that, data is portioned into the training and testing phase. Furthermore, we apply CNN to extract features from it. After the training is completed, the test dataset is used for validation. The prediction accuracy is calculated based on the model's performance in the validation phase.

### 2.2. Generation of Spectrogram

The spectrogram refers to representing the frequencies on the image that are present on a signal over time. The signal's frequency gives rise from a time series signal of data points using Fast Fourier Transform (FFT). Fast Fourier Transform (FFT) can be put into time-series data to calculate the magnitude of the frequency for a fixed moment in time. The process of time-series data is first windowed, usually in small chunks, and the FFT data is kept together to form the spectrogram images, which empowers us to see how fast the frequencies improve.

Since the work was done to generate spectrograms on audio clips or utterances of data, then data was regenerated into Mel spectrograms, known as spectrograms images. The conversion frequencies from *f* hertz type to *m* mels are shown in Figures 3 and 4:

(1) $$\begin{array}{c} m=2595\;\log_{10}\left(1+\frac{f}{700}\right). \end{array}$$

### 2.3. Bernoulli Naïve Bayes

Bernoulli Naïve Bayes uses discrete data and it works on Bernoulli distribution. The main feature of Bernoulli Naïve Bayes is that it accepts features only as binary values like true or false, yes or no, 0 and 1, success or failure, and so on. As they deal with binary values, let us consider ‘*p*' as the probability of success and ‘*q*' as the probability of failure and *q* = 1 − *p*, for a random variable ‘*X*' in Bernoulli distribution:

(2) $$\begin{array}{c} p\left(x\right)=P\left[X=x\right]=\left\{\begin{array}{cc} q=1-p, & x=0,\\ p, & x=1, \end{array}\right) \end{array}$$

where ‘*x*' is in binary form like 0 or 1. The Bernoulli Naïve Bayes machine learning classifier is based on

(3) $$\begin{array}{c} p\left(x_{i}|y\right)=P\left(i|y\right)x_{i}+\left(1-P\left(i|y\right)\right)\left(1-x_{i}\right). \end{array}$$

## 3. Related Work

Literature [15] proposed a deep learning-based spoken language identification system. It combines DNNs and *i*-vectors to increase efficiency. Every hidden layer includes 2560 neurons with a ReLU function. They use the softmax activation function in the last layer. It compares a DNN and *i*-vectors on two different datasets: LRE′09 and Google 5M lid corpus. With these two approaches, they failed to achieve good results. They also compare the performance with Equal Error Rate (EER), where they got an average of 9.58% using the DNN model. Literature [16] proposed a method that can improve generalization to identify short speech-language using triplet entropy loss with the help of CNN; they combine cross-entropy loss (CEL) and triplet loss through which they generalize the data and use it on Slavic languages. They use ResNet50 pretrained model and use the softmax function at the last layer. It uses an Adam optimizer with the learning rate (LR) of 10e-4, uses the batch size of 32, and ridge-based regularization to reduce overfitting. The top accuracy they achieved was 78% using triplet loss. They showed Triplet Entropy loss is better than cross-entropy loss, but they failed to achieve good performance.

Literature [17] proposed an unsupervised neural-based model which can be used in spoken language identification and can decrease the distribution variance on both attributes and classifiers for the training and testing datasets. It proposed the optimal transport (OT) method to measure the distribution of the discrepancy. The Time Delay Neural Network (TDNN) framework is used for determining training and test set adaption. Literature [18] proposed a deep neural network-based model which identifies a Slavic language or those languages which are similar. They created the model with two parameters: segment level feature extractor and language classifier. The model uses the CNN with 128, 256, and 512 filters with 5, 10, and 10 for each layer with stride 1 at each layer. They use two techniques, Baseline LID and Robust LID. In baseline LID, they got 53.25 as average accuracy, and in robust LID, they got 87.32 as average accuracy. Literature [19] proposed a framework that combines CNN and LSTM system that uses CTC loss function to train the model. In this, audio clips are converted into spectrograms, further CNN is applied to extract the features from it, and further LSTM is used to store the data from previous layers. The speech signal is sampled at 16 KHz with window size 200 ms, and window stride with 100 ms. This method gives an accuracy between 74% to 76%.

Literature [20] proposed a capsule network framework for identifying spoken language identification systems. In CapsNet, a convolutional layer has a total of 128 kernels with the size of (9,9,1) and a step size of 1 with ReLU function. It divided the CapsNet into two parts: encoder and decoder. The first 4 layers represent the encoder, and the last 3 layers represent the decoder. They achieved an accuracy of 91.80% with 5-second audio clips using the CapsNet approach. Literature [21] proposed various feature selection methods like top-*k* selection, forward feature selection, and recursive feature elimination, so the model can work efficiently. In the first phase, preprocessing is done in which it removes the punctuations, emoticons, links, hashtags, URLs, then removes the less important words using the English stop words, and then removes redundant data from the dataset. The top-k feature method performs well; it selects 550 features compared to the other methods. Literature [22] proposed a Recurrent Neural Network Transducer (RNN-T) for speech recognition and spoken language identification. They use two languages pair: English-Spanish and English-Hindi. The RNN-T framework uses 5 encoder LSTM layers with 1024 units and 2 decoder LSTM layers with 1024 units; a 512-d embedding layer was used as a decoder input. The discrete fracture network (DFN) has 512 hidden neurons, along with tanh and softmax functions.

Literature [23] proposed a technique that associates with acoustic level representations with embedding on Automatic Speech Recognition, which gives a 50% reduction in error rate. They used 64-d log-Mel feature extractors for training on a 25 ms window with a 10 ms overlap. The first 3 LSTM layers comprise 768 units, and all the data is further passed to FC layers and softmax function. At last, they used a semisupervised technique to increase the accuracy and good results of the model. Literature [24] proposed a signal combination approach for language identification. They used a deep learning model to combine the signals from recognizers with the baseline, which uses low-level acoustic signals. It helps to decreases the error rate from 5.50% to 4.30%. They work with 11 different models and use ReLU, dropouts, Adam, batch normalization, and various other attributes to get good results. Literature [25] proposed a system with an acoustic model and a context-aware model. They created the model with 4 convolutional layers with 128 units, 4 fully connected layers with the 1024 units, 1 fully connected layer with the 512 units, 1 temporal pooling layer with a mean and standard deviation, 1 fully connected layer with 1024 units, and at last softmax function is used with unit 1. With this framework, they got 97.0% accuracy. Literature [5] proposed a conditional GANs classifier framework for language identification, choosing GANs is a better option on large datasets, giving good results. 2 × 2 is used to perforate upsampling, 5 × 5 Conv. 1, tanh, and an output (49) tanh is used. With this framework, they achieved 97% accuracy.  Table 1 summarizes the previous studies, features, and results as discussed above.

## 4. Proposed Spoken Language Identification Framework

This section discusses the motivation and the spoken language identification framework.

### 4.1. Motivation

Various state-of-the-art results on various audio classification tasks have been obtained by using log-Mel spectrograms of raw audio, like features, which convert the audio utterance into images [8]. CNN gives an excellent performance gain in classification on these features [14]. The motivation of work has come from these studies. The computation time is more for converting audio into spectral images, giving us a new direction to develop the computationally efficient and more accurate spoken identification technique.

### 4.2. Proposed Spoken Identification Framework

The proposed deep learning-based spoken language identification framework: while designing this framework, audio utterances are converted into spectrograms based on their frequency and time. After this, a convolutional neural network (CNN) is applied to images to extract their features for classification. At last, the softmax activation function is applied for multilanguag classification.

### 4.3. Preprocessing

In the preprocessing phase, data augmentation is used to solve class imbalance problems. Data augmentation reduces overfitting and acts as a regularizer when training a model. With the help of data augmentation, it can increase the amount of data by adding some modifications of existing data like crop, rotate, flip, shearing, and much more effects. The use of data augmentation is good while using transfer learning models works well on more data and predicts good results.

### 4.4. Description of Features

The duration of each audio is 10 seconds (sharp) with a sample rate of 22050, a bit depth of 16 bits, and channels 1, and each audio file is a Free Lossless Audio Codec (FLAC) audio sample. The dataset is divided into two directories: *train,* which contains (73080) samples, and *test,* which contains (540) samples, with three languages English, German, and Spanish. Several audio transformations are applied, like pitch, speed, and noise. It contains the voice of 90 original speakers of male and female.

### 4.5. Model Description

In the model description, it describes the framework to all the models for the experiment purpose:

- An appropriate pooling layer always follows every convolutional layer. It helps to include the explosion of attributes and keeps the model small and efficient.
- Each convolution layer is followed by the dropout layer, ReLU, and batch normalization. The batch normalization is responsible for the convergence of learned representations.
- Finally, a dense layer is used, which acts as an output layer of the model.

### 4.6. Model Characteristic: 2D ConvNet

Table 2 presents a specific layer-by-layer explanation of the model with its different hyperparameters.

### 4.7. Model Characteristic: Word Embedding

Table 3 presents a layer-by-layer explanation of the model and the details of hyperparameters.

The above word embedding model is a pretrained model by Keras use for experiments for language identification. The first step is to download the stop words using the *nltk* library; after that, there are 22 languages in the dataset like Arabic, Chinese, Dutch, English, Estonian, French, Hindi, Indonesian, Japanese, Romanian, Korean, Latin, Persian, Portuguese, Pushto, Russian, Turkish, Swedish, Tamil, Thai, Urdu, and Spanish. Each language contains 1000 rows in the dataset. After completing the preprocessing, then further divide the data into the train and test set. Then, apply the word embedding model to the dataset at the output layer; softmax is used because there are 22 classes. With this model, the achieved accuracy is 95%.

### 4.8. Model Details: Bernoulli Naïve Bayes

This approach uses the Bernoulli Naïve Bayes machine learning technique to identify language from a given dataset. In a preprocessing step, all the data are first split into *X* and *Y* and then encode the data using a label encoder library. Following that, perform data cleaning to convert all the sentences into lower case. Then, the Naïve Bayes approach is applied, which takes 29.7 seconds to fit in the model and gives me 93.0% accuracy.  Table 4 shows the metrics that are performed using Naïve Bayes.

## 5. Experimental Results and Discussion

This section contains results and a discussion of different techniques. All the details regarding the use of datasets, hyperparameter settings, evaluation metrics, and computational time analysis of the different proposed approaches are illustrated.

### 5.1. Datasets

The experiment of the different techniques is implemented using the four datasets, spoken language identification [30], language identification dataset [31], common voice Kaggle [32], and Mozilla common voice dataset [33], which are described in Table 5.

Spoken language identification [30] dataset consists of 73080 train samples and 540 test samples with three languages: English, German, and Spanish. It contains both male and female recordings. The audio files have Free Lossless Audio Codec (FLAC) extensions. Language identification [31] dataset consists of 22000 train samples with 22 languages: Arabic, Chinese, Dutch, English, Estonian, French, Hindi, Indonesian, Japanese, Korean, Latin, Persian, Portuguese, Pushto, Romanian, Russian, Spanish, Swedish, Tamil, Thai, Turkish, and Urdu. All data is stored in a CSV file with 1000 rows per language. Common voice Kaggle [32] dataset consists of 354785 audio samples, which are further divided into six folders with 16 main languages: United States English, Australian English, England English, Canadian English, Filipino, Hong Kong English, India, and South Asia, Irish English, Malaysian English, New Zealand English, Scottish English, Singaporean English, South Atlantic, South African, Welsh English, West Indies, and Bermuda; all languages are stored as mp3 files. It contains both male and female recordings. Mozilla common voice [33] dataset contains four languages, Estonian, Tamil, Turkish, and Mandarin, to check the robustness of the model. It includes 23842 audio samples, which are further divided into train samples and test samples. It contains both male and female recordings. This dataset is available in both audio clips and TSV files.

### 5.2. Hyperparameter Details

The attributes of the proposed method are represented in Table 6. The trial and error method is used while running the convolution neural network [8, 14], word embedding Keras [34, 35], and Naïve Bayes [36–38]. The selection of hyperparameter is also defined as an NP-complete problem [39, 40]. The efficient selection of hyperparameters can achieve better results [41, 42]. In CNN, the epochs are set to be 60, and the size of the batch is 32 with ReLU as an activation function. Dropouts [43, 44] are used with Adam optimizer. At the output layer, the softmax function [45] is used. In word embedding, it is a pretrained model by Keras. It is used in which the epochs are 25, and categorical cross-entropy loss is applied with Adam optimizer. Bernoulli naïve Bayes classifier is implemented with kernel function Bernoulli.

### 5.3. Performance Evaluation Metrics

The evaluation metrics are used for experimentation to check the performance of the model. Those are precision, recall, F1 score, and accuracy as shown in Table 7.

A receiver operating characteristic (ROC) curve is a graph that represents the classification model at different classification threshold values. These curves plot two parameters or attributes of ROC: false positive rate (FPR) and true positive rate (TPR).

In Figure 5, a multiclass ROC curve for language identification is presented. This spoken language identification Kaggle dataset contains three languages: German, English, and Spanish. Similarly, the ROC curve is also made like this for the language identification Kaggle dataset, which contains 22 languages: English, Arabic, French, Hindi, Urdu, Portuguese, Persian, Pushto, Spanish, Korean, Tamil, Turkish, Estonian, Russian, Romanian, Chinese, Swedish, Latin, German, Dutch, Japanese, and Thai.

## 6. Results and Discussion

The presented work discusses various methods which attain state-of-the-art results using four different datasets with audio, and the first dataset contains three languages, the second dataset includes 22 languages, and the third dataset includes 16 languages. All are available on the Kaggle and fourth Mozilla common voice dataset contains four languages and is available on the Mozilla website. In the image domain, 2D convolutional neural networks obtained an accuracy of 98%. In another dataset of CSV file, word embedding using the pretrained model obtained an accuracy of 95%. With Bernoulli Naïve Bayes approach, we obtained an accuracy of 93% on a 22-language dataset. Using the SVM and random forest classifier model achieved 82.88% and 72.42% accuracy on the 16-language dataset.

### 6.1. Misclassification

Various languages in the world belong to the Indo Persian and European families. In this group, the languages are separated into three subparts: Germanic, Romance, and Slavic. Our model confuses those languages with the same words; for example, “Cat” word in English, “Chatte” word in French, “Kat” word in Dutch, and “Katze” in German all have the same sound and pronunciation; hence, it is very difficult for a model to understand. Our model confuses Russian (Ru) and French (Fr) because they have similar accents; many words are adopted from French to Russian, so it is very difficult to give accurate results.

### 6.2. Performance of Classification Model: Confusion Matrix

In this section, the performance of the model is shown in Figure 6, using a confusion matrix for multiclass classification representing three classes of English, Spanish, and German. In this matrix, diagonal elements are predicted the same as the true value while nondiagonal elements are not classified properly by the model. On the *x*-axis, there is the true label, and on the *y*-axis, there is a predicted label.

In Figure 6, the multiclass confusion matrix for language identification in this spoken language identification Kaggle dataset is used, which contains three languages: German, English, and Spanish. Similarly, the confusion matrix is also made like this for the language identification Kaggle dataset, which includes 22 languages: English, Arabic, French, Hindi, Urdu, Portuguese, Persian, Pushto, Spanish, Korean, Tamil, Turkish, Estonian, Russian, Romanian, Chinese, Swedish, Latin, German, Dutch, Japanese, and Thai.

### 6.3. Performance Evaluation

Table 8 represents the performance comparison of various spoken language identification techniques using CNN, Naïve Bayes, word embedding, SVM, logistic regression, VGG16, ResNet50, and, random forest classifier. Spoken language identification contains three languages with train and test folders which include audio clips of different languages. Using CNN, the accuracy obtained 100% with good results and better achieved better precision, recall, and F1 score. The language identification dataset contains 22 languages in a CSV file which contains multiple sentences of each language. By using Naïve Bayes and word embedding techniques, the accuracy obtained 94% and 95% but is less efficient than the CNN technique. The Common voice Kaggle dataset contains 16 languages using SVM and random forest classifier techniques. The accuracy achieved is 82.88% and 72.42%, which is good enough. The Mozilla common voice dataset contains four languages using VGG16 and logistic regression techniques. The accuracy obtained was 81.30% and 84.30 with good results.

### 6.4. Convergence for Training and Validation

This section is basically on the use of various optimizers on train and validation accuracy to compare our model. In Figure 7(a), the RMSprop optimizer with five epochs gives good results. In Figure 7(b), the use of Nadam optimizer with five epochs and its performance is not so good as compared to other optimizers. In Figure 7(c), the use of an SGD optimizer with five epochs and performance is a little bit better than the Nadam optimizer. In Figure 7(d), the use of Adam optimizer with five epochs also works well and gives good results.

## 7. Conclusion and Future Scope

There are two contributions of the paper in the field of spoken language identification. Firstly, we use the deep learning architecture for image classification in identifying languages from generated images from audio. Powerful performance can be achieved using relatively short files with minimum preprocessing. We believe that this model can be extended to more languages as long as sufficient. This approach achieved an accuracy of 98% and gave us good results. Secondly, we use the Bernoulli Naïve Bayes approach on a language identification dataset with 22 languages. It takes a little bit more time as compared to CNN in model fitting data. This approach gives us an accuracy of 93%. And further, we apply another approach to this dataset, a pretrained model by Keras that is word embedding. It is a little bit faster and more accurate than Naïve Bayes. This approach achieved an accuracy of 95%.

The performance of log-Mel spectrograms can be additionally refined by removing the noise from audio. There is a possibility for improvement by data augmentation on the available data using different methods like pitch shifting, crop, rotate, flip, adding random noise, and changing audio speed, and various methods. These help in making neural networks more robust to modifications that might be present in real-world scenarios. There is often further observation or review of various feature extraction techniques like Constant-Q transform and Fast Fourier Transform and their impact on language identification. These are known to possess a positive impact on the performance of convolutional neural networks.

## Figures and Tables

**Figure 1:** Schematic diagram of the spoken language identification system.

**Figure 2:** Phases of spoken language identification using spectrograms.

**Figure 3:** Generated spectrogram from an English audio file.

**Figure 4:** Wavelength of audio.

**Figure 5:** ROC curve.

**Figure 6:** Confusion matrix for the multiclass spoken language identification.

**Figure 7:** Use of different optimizers for comparison.

**Table 1:** Review of previous studies along with results.

Year	Model basis	Features	Languages	Acc.	Remarks	Ref.
2021	PLDA logistic regression	*i*-vector *x*-vector	Javanese, Sundanese, Minang	96%	PLDA and logistic classifiers are used with *x*-vector and *i*-vector feature extraction.	[26]
2021	CNN ResNet50 RNN	MFCC	Iba, Kab, Sun, Ind, Eus, Jav, Tam, Tel, Kan, Hin, Tha, Rus, Cnh, Eng, Por, Mar	53%	Submit three different systems named Lipsia, Anlirika, and NTR with different specifications.	[27]
2021	Self-attentive pooling decoder	Not defined	En, Fr, Es, De, Ru, It	92.50%	Used self-attentive pooling layer for language identification task.	[28]
2021	CNN LSTM	MFCC	Iba, Kab, Sun, Ind, Eus, Jav, Tam, Tel, Kan, Hin, Tha, Cnh, Eng, Por, Mar, Rus	74%	CNN-LSTM combination is used for predicting language.	[29]
2020	TDNN optimal transport	MFCC	Russian, Kazakh, Mandarin, Korean, Japanese, Cantonese, Vietnamese, Tibetan, Indonesian, Uyghur	Not defined	Used unsupervised technique joint distribution adaptation neural network model for spoken language identification.	[17]
2020	CRNN ResNet50 DenseNet121	Log-Mel	Three different datasets with different languages	89%	Used different pretrained models with triplet entropy loss for improving the generalization.	[16]
2020	CNN	Log-Mel	Slovene, Russian, Slovak, Belarusian, Macedonian, Ukrainian, Croatian, Bulgarian, Czech, Serbian, Polish	97.35%	With the CNN model, two neural models are made: baseline and robust models for spoken language identification.	[18]
2020	CapsNet	Log-Mel	Arabic, Bengali, Chinese Mandarin, English, Hindi, Turkish, Spanish, Japanese, Punjabi, Portuguese	98.20%	Capsule network with encoder and decoder works well on spoken language identification.	[20]
2020	CNN-LSTM	Log-Mel	Gujarati, Tamil, Telugu	79.02%	Used CNN-LSTM system that uses CTC loss function at output layer and this approach is used for spoken language identification.	[19]
2020	Context aware model	Log-Mel	Prs, Amh, Fas, Hat, Hau, Eng, Cmn, Fra, Rus, Hin, Ukr, Spa, Pus, Urd, Yue, Bos, Vie, Hrv, Tur, Kat, Por, Kor	97%	Context-aware model works well on pair language and gives good results and better accuracy.	[25]
2019	ConvNets	MFCC	Fr, It, En, Ru, Es, De	95.40%	2D ConvNets with attention and GRU approach gives good results and better accuracy.	[14]
2019	ResNet50	MFCC	Fr, It, En, Ru, Es, De	89%	In this, used pretrained ResNet50 model and cyclic learning rate approach for language identification.	[8]
2018	SVM-HMM model	Not defined	Es, Fr, En, De	70%	In this, HMMs approach was used to translate speech into the vector sequences following the deep neural network.	[30]
2017	Inceptionv3 CRNN	MFCC	Es, De, En, Fr	96%	The pipeline of inception-v3 based transfer learning and bi-LSTM was used to extract temporal and convolutional attributes.	[24]
2010	Gaussian mixture model	Perceptual linear prediction	Tel, Dut, Hi, En, Ben, Fr, Es, De, Ru, It	88.80%	The use of Gaussian mixture models with the RPLP approach, which are processed using PLP and MFCC features.	[3]
2009	CNN-TDNN	MFCC	Fr, De, En	91.20%	Log-Mel images were used as features for language identification coupled with SGD based neural network.	[2]

**Table 2:** Architecture of 2D ConvNet model.

Layers	Filters, kernels, and stride	Padding	Output	No. of parameters
First block				
Conv2D	(32, 7, 7)	Valid	(None, 994, 34, 32)	1600
BatchNorm			(None, 994, 34, 32)	128
MaxPool2D	(3, 3) *s* = 2	Same	(None, 497, 17, 32)	0
Second block				
Conv2D	(64, 5, 5)	Same	(None, 497, 17, 64)	51264
BatchNorm			(None, 497, 17, 64)	256
MaxPool2D	(3, 3) *s* = 2	Same	(None, 249, 9, 64)	0
Third block				
Conv2D	(128, 3, 3)	Same	(None, 249, 9, 128)	73856
BatchNorm			(None, 249, 9, 128)	512
MaxPool2D	(3, 3) *s* = 2	Same	(None, 125, 5, 128)	0
Fourth block				
Conv2D	(256, 3, 3)	Same	(None, 125, 5, 256)	295168
BatchNorm			(None, 125, 5, 256)	1024
MaxPool2D	(3, 3) *s* = 2	Same	(None, 63, 3, 256)	0
Fifth block				
Conv2D	(512, 3, 3)	Same	(None, 63, 3, 512)	1180160
BatchNorm			(None, 63, 3, 512)	2048
MaxPool2D	(3, 3) *s* = 2	Same	(None, 32, 2, 512)	0
Flatten layer			(None, 32768)	0
BatchNorm			(None, 32768)	131072
Dense layer	256		(None, 256)	8388864
BatchNorm			(None, 256)	1024
Dropout	0.5		(None, 256)	0
Dense layer	3		(None, 3)	771

**Table 3:** Architecture of word embedding model.

Layers	Output	No. of parameters
Embedding layer	(None, 100,500)	136984000
Flatten	(None, 50000)	0
Dense layer	(None, 22)	1100022

**Table 4:** Evaluation metrics using the Bernoulli Naïve Bayes model.

Evaluation metrics	Score
Precision	0.946460
Recall	0.931159
F1 score	0.931159
Matthews correlation coefficient	0.925470

**Table 5:** Dataset description.

Dataset	Spoken language identification [30]	Language identification dataset [31]	Common voice Kaggle dataset [32]	Mozilla common voice dataset [33]
Number of languages	3	22	16	4
Total samples	Train = 73080 (420 mins) Test = 540 (90 mins)	22000	354785	23842
Type	Audio	Text	Audio	Audio and TSV
Length	10 seconds	7 to 10 sentences in each line	Less than 10 seconds	Less than 10 seconds
Extension	FLAC	CSV	Mp3	Mp3 and TSV

**Table 6:** Parameter setting.

Proposed technique/parameters	Value
Convolutional neural network	
Number of epochs	60
Batch size	32
Activation	ReLU
Optimizer	Adam
Dropouts	Yes
Loss	Categorical cross-entropy
Activation output	Softmax
Word embedding	
Number of epochs	25
CNN model	Word embedding Keras
Loss	Categorical cross-entropy
Optimizer	Adam
Activation output	Softmax
Naïve Bayes	
Type	Bernoulli Naïve Bayes
Kernel function	Bernoulli

**Table 7:** Different evaluation metrics.

Sr. no.	Metrics	Equation	Remarks	Ref.
1	Accuracy (acc)	(*tp*+*tn*/*tp*+*fp*+*tn*+*fn*)	It is the ratio of correct outputs compared to the total number of outputs.	[30]
2	Precision (p)	(*tp*/*tp*+*fp*)	It is the ratio of correct positive predictions from the total prediction from the positive class.	[30]
3	Recall (r)	(*tp*/*tp*+*tn*)	The recall is used to measure the fraction of positive patterns that are correctly classified.	[30]
4	F1 score (FM)	(2^*∗*^*p*^*∗*^*r*/*p*+*r*)	The F1 score refers to or represents the harmonic mean between recall and precision values.	[30]

**Table 8:** Performance measures obtained from various language identification techniques.

Models	Dataset used	Train acc.	Test acc.	Validation acc.	Sensitivity	Specificity	F1 score	Precision	Recall
CNN	Spoken language identification	100	98.63	98.90	98.90	99	99.90	99.90	99.90
Naïve Bayes	Language identification dataset	94	94	93	100	99	93.60	94.90	93.60
Word embedding	Language identification dataset	95.50	92.20	93.20	98	99	92.50	93.50	92.50
Logistic regression	Spoken language identification	64.32	61.95	63.55	64.23	63.55	64.23	64.23	64.23
Naïve Bayes	Spoken language identification	50.25	49.75	51.20	52.32	51.78	51.20	51.20	51.20
SVM	Common voice Kaggle	82.88	83.32	82.65	75.95	75.55	76.95	76.95	76.95
Random forest classifier	Common voice Kaggle	72.42	71.90	71.50	66.32	67.24	67.23	67.23	67.23
VGG16	Mozilla common voice	81.30	80.21	81.05	81.25	80.52	79.83	80.02	80.02
ResNet50	Spoken language identification	86.30	80.20	84.32	85.36	84.23	84.65	82.75	82.75
CapsNet [20]	Spoken language identification	91.80	88.76	90.72	88	89	89	89	89
2D ConvNet bidirectional GRU [14]	Spoken language identification	68.85	65.23	67.82	68	66	66	66	66
Acoustic model [25]	Spoken language identification	75.69	73.23	74.23	75	75	75	75	75
CNN LSTM [19]	Spoken language identification	83.25	80.52	82.45	83	82	82	82	82
Logistic regression I-vector [26]	Mozilla common voice	84.30	80.23	82.52	78.95	80.05	82.36	82.36	82.36
LSTM-CNN [29]	Common voice Kaggle	70.21	68.33	69.96	67.23	68.33	69.54	69.54	69.54

## Data Availability

The data that support the findings of this study are available upon request.
